# Monocrotophos Induces the Expression and Activity of Xenobiotic Metabolizing Enzymes in Pre-Sensitized Cultured Human Brain Cells

**DOI:** 10.1371/journal.pone.0091946

**Published:** 2014-03-24

**Authors:** Vinay K. Tripathi, Vivek Kumar, Abhishek K. Singh, Mahendra P. Kashyap, Sadaf Jahan, Ankita Pandey, Sarfaraz Alam, Feroz Khan, Vinay K. Khanna, Sanjay Yadav, Mohtshim Lohani, Aditya B. Pant

**Affiliations:** 1 In Vitro Toxicology Laboratory, CSIR-Indian Institute of Toxicology Research, Lucknow, India; 2 Metabolic and Structural Biology Department, CSIR-Central Institute of Medicinal and Aromatic Plants, Lucknow, India; 3 Department of Biotechnology, Integral University, Lucknow, India; CSIR-Central Drug Research Institute, India

## Abstract

The expression and metabolic profile of cytochrome P450s (CYPs) is largely missing in human brain due to non-availability of brain tissue. We attempted to address the issue by using human brain neuronal (SH-SY5Y) and glial (U373-MG) cells. The expression and activity of CYP1A1, 2B6 and 2E1 were carried out in the cells exposed to CYP inducers viz., 3-methylcholanthrene (3-MC), cyclophosphamide (CPA), ethanol and known neurotoxicant- monocrotophos (MCP), a widely used organophosphorous pesticide. Both the cells show significant induction in the expression and CYP-specific activity against classical inducers and MCP. The induction level of CYPs was comparatively lower in MCP exposed cells than cells exposed to classical inducers. Pre-exposure (12 h) of cells to classical inducers significantly added the MCP induced CYPs expression and activity. The findings were concurrent with protein ligand docking studies, which show a significant modulatory capacity of MCP by strong interaction with CYP regulators-CAR, PXR and AHR. Similarly, the known CYP inducers- 3-MC, CPA and ethanol have also shown significantly high docking scores with all the three studied CYP regulators. The expression of CYPs in neuronal and glial cells has suggested their possible association with the endogenous physiology of the brain. The findings also suggest the xenobiotic metabolizing capabilities of these cells against MCP, if received a pre-sensitization to trigger the xenobiotic metabolizing machinery. MCP induced CYP-specific activity in neuronal cells could help in explaining its effect on neurotransmission, as these CYPs are known to involve in the synthesis/transport of the neurotransmitters. The induction of CYPs in glial cells is also of significance as these cells are thought to be involved in protecting the neurons from environmental insults and safeguard them from toxicity. The data provide better understanding of the metabolizing capability of the human brain cells against xenobiotics.

## Introduction

The key role of cytochrome P450s (CYPs) super-family in endogenous and xenobiotic metabolism is well established [1], [2]. Though the liver has been reported as the major CYPs mediated metabolic site [3], but the significant expression and activity of selected CYPs has also been reported in brain tissues [4], [5], [6]. In general, the brain has a comparatively lower level of expression and activity of CYPs than liver, but due to tissue heterogeneity few specific regions and cells of the brain have been reported to have significantly higher expression and activity of CYPs than that of liver [7], [8]. The regional specific expression and inducibility of several members of the CYP gene family involved in metabolism, toxicity and detoxification have already been documented in the brain of experimental animals receiving exposure to environmental chemicals and drugs [4], [9]. Brain cells have shown high inducibility of CYPs, and quite often in a different fashion from their hepatic forms [10], [11]. Our group has also shown the constitutive and inducible expression of CYPs in human and rat brain primary culture of neuronal and glial cells [12], [13], [14], [15]. Immortalized human-derived brain endothelial cell line has also reported to express CYP enzymes [16], [17].

CYPs in families 1 to 3 are primarily involved in the detoxification of various xenobiotic compounds and drugs [18], whereas the remaining groups are broadly play the role in the metabolism of endogenous compound such as steroids, fatty acids, hormones, neurotransmitters, cholesterol, bile acids and vitamins, etc. [19]. Khokhar and Tyndale [20] provided strong evidences supporting the role of brain CYPs in local drug metabolism, and subsequent alterations in the pharmacological actions of drugs. CYP1A1 is well known for its role in the bioactivation of carcinogens such as aromatic amines and polycyclic aromatic hydrocarbons (PAHs) [21], [22]. Induction and a high activity of the CYP1A1 have been associated with increased toxicity and cancer risk [23], [24]. CYP2B6 is also expressed in the brain, highly expressed in specific cells such as cortical pyramidal cells and astrocytes [25] and may be an important factor in the metabolism of drugs acting on the central nervous system (CNS). The concentration of CYP2B6 in the brain regions of smokers and alcoholics has been reported abnormally high, particularly in the cerebellar Purkinje cells, granular cell layer and hippocampal pyramidal neurons [26]. CYP2B6 metabolizes a wide range of substances including endogenous compounds such as arachidonic acid, 17 β-estradiol, testosterone [27] and the neurotransmitter serotonin [28], dopamine [29] and neurotoxins [30]. It metabolizes therapeutically important drugs as well as drugs of abuse [31], [32]. The expression of CYP2E1 has also been reported in cultured rat [13], [33] and human brain cells [34]. The mechanism of CYP2E1 induction is complex and depends on the substrate, species, tissue, or cell type [35], [36] and in the brain regions and cell type specific expression [37]. CYP2E1 enzymes are involved in the metabolism of alcohol other low-molecular-weight xenobiotics, including drugs, organic solvents, and pro-carcinogens [38], [39], [40]. CYP2E1 have potential impact on brain function by metabolizing ethanol resulting in generation of reactive oxygen species that have direct concern in the neurodegenerative disorders such as Parkinson's disease, minor dendritic and synaptic changes to neuronal cell death [41], [42] through lipid peroxidation, protein inactivation, and DNA damage [43]. The protein level of CYP2E1 in smokers has significantly more in comparison to non-smokers in several brain regions [7], [44].

Inspite of several investigations pertaining to the metabolizing capabilities of CYPs in brain tissues and primary cultures of brain cells of experimental animals, the status of these CYPs in human brain cells is poorly understood. The reason being is non-availability of human brain due to ethical dubious. Thus, to address the issue, the expression and inducibility of CYP1A1, CYP2B6 and CYP2E1 were investigated in cultured human brain neuronal (SH-SY5Y) and glial (U373-MG) cell lines. Xenobiotic metabolizing capability of cells was studied using known inducers of CYP1A1 (3-methylcholanthrene), CYP2B6 (cyclophosphamide) and CYP2E1 (ethanol). The studies were further extended to investigate the responsiveness of CYPs in the cells against monocrotophos, a widely used organophosphate pesticide used in many parts of the world, including India for more than forty years and known for its systemic toxicity including neurotoxicity [45], [46], [47].

## Materials and Methods

### Reagents and Consumables

All the specified chemicals and reagents *viz.*, monocrotophos (MCP), 3-methylcholanthrene and cyclophosphamide (CPA) were purchased from Sigma (Sigma St Louis, MO, USA) unless otherwise stated. Culture medium DMEM/F-12, antibiotics, fetal bovine serum and Trypsin-EDTA were purchased from Gibco BRL, USA. All the antibodies used in this study were procured from Chemicon International, USA. Culture wares and other plastic wares used in the study were procured commercially from Nunc, Denmark. Milli Q water (double distilled, deionized water) was used in all the experiments.

### Cell Culture

Human neuroblastoma cell line SH-SY5Y and glioblastoma U373-MG cell lines used in the study were initially procured from National Centre for Cell Sciences, Pune, India and since then have been maintained at In Vitro Toxicology Laboratory, Indian Institute of Toxicology Research, Lucknow, India, as per the standard protocols. In brief, the cells were cultured in DMEM/F-12, supplemented with 10% fetal bovine serum (FBS), 0.2% sodium bicarbonate, 100 units/ml penicillin G sodium, 100 µg/ml streptomycin sulfate and 0.25 µg/ml amphotericin B. Cultures were maintained at 370C, in 5% CO_2_-95% atmosphere under high humid conditions. Medium was changed twice weekly and cultures were passaged at a ratio of 1∶6 once in a week. Prior to use in the experiments, cell viability was ascertained by Trypan blue dye exclusion assay. The culture showing viability more than 95% were used in all the experiments. All the experiments were done on the cells with passage 18–25 only.

### Identification of non-cytotoxic doses of MCP, 3-MC, CPA and Ethanol

In the present investigations, known inducers of CYP1A1 [3-methylcholanthrene (3-MC)], CYP2B6 [cyclophosphamide (CPA)], CYP2E1 [ethanol] and known neurotoxin - monocrotophos (MCP), an organophosphate pesticide, were used. 3-MC was dissolved in culture grade dimethylsulphoxide (DMSO), while CPA, ethanol and MCP were dissolved in DMEM/F-12 medium. Prior using in the expression studies, non-cytotoxic doses of 3-MC, CPA, ethanol and MCP were identified in SH-SY5Y (human neuronal cell line) and U373-MG (human glial cell line). Cytotoxicity assessment was done using standard endpoint i.e., tetrazolium bromide MTT (3-(4, 5-dimethylthiazol-2-yl) -2, 5-diphenyl tetrazolium bromide) assay as described earlier by us [48]. In brief, neuronal - SH-SY5Y cells and glial - U373-MG cells (1×10^4^ cells/well) were seeded in 96-well tissue culture plates and incubated in the CO_2_ incubator for 24 h at 37°C. Then the medium was aspirated and cells were exposed to medium containing either of 3-MC (1 µM–10 µM), CPA (0.5 mM–8 mM), ethanol (25 mM–400 mM) and MCP (10^−7^ M–10^−3^ M) for 24–96 h at 37°C in 5% CO_2_-95% atmosphere under high humid conditions. Tetrazolium salt (10 µl/well; 5 mg/ml of stock in PBS) was added 4 h prior to completion of respective incubation periods. At the completion of incubation period, the reaction mixture was carefully taken out and 200 µl of culture grade DMSO was added to each well. The content was mixed well by pipetting up and down several times until dissolved completely. Plates were then incubated for 10 minutes at room temperature and color was read at 550 nm using Multiwell Microplate Reader (Synergy HT, Bio-Tek, USA). The unexposed sets, and sets exposed to MnCl_2_ (10^−4^ M) were also run parallel under identical conditions that served as a basal and positive control respectively.

### Experimental Design

The flow map of experimental design is depicted in Figure 1.

**Figure 1:** Experimental design of the study.

### Transcriptional Changes

Transcriptional changes in the selected CYPs (1A1, 2B6 and 2E1) were studied in both neuronal and glial cell lines exposed to various concentrations of CYP inducers and pesticide-monocrotophos as described in experimental design. Xenobiotics induced alterations in the mRNA expression level were expressed in relative quantification by comparing the data obtained from unexposed cells. The quantitative Real Time PCR analysis was done following the protocol described earlier by us [49]. In brief, total RNA was isolated from both experimental and unexposed control sets using Gene Elute mammalian total RNA Miniprep Kit (Catalog No. RTN-70, Sigma, USA). Total RNA (1 µg) was reverse transcribed into cDNA by Super Script III first strand cDNA synthesis kit (Catalog No. 18080-051, Invitrogen Life Science, USA). Quantitative real time PCR (RT-PCRq) assay reactions were carried out with 2× SYBR Green PCR master mix (Applied Biosystems, USA) using ABI PRISM 7900HT Sequence Detection System having software version 2.2.1 (Applied Biosystems, USA). Results were expressed relative to the housekeeping gene i.e., β-actin. Real time reactions were carried out in triplicate wells for each sample. The gene specific primers used were as follows: β-actin sense, 5′-aaccccaaggccaaccg-3′; β-actin antisense, 5′-agggatagcacagcctgga-3′ [50]; CYP1A1 sense, 5′-accttccgacactcttccttcg-3′; CYP1A1 antisense, 5′-cagatgggttgacccatagcttct-3′ [50]; CYP2B6 sense, 5′-tggaggatggtggtgaagaag-3′; antisense, 5′-tgccatcaaggataggcaag-3′ and CYP2E1 sense, 5′-tgccatcaaggataggcaag-3′; antisense, 5′-caacaaaagaaacaactccatga-3′ (designed with Primer Express 3.0 software; Applied Biosystems, USA).

### Translational changes (Western Blot Analysis)

Translational changes in the selected CYPs (1A1, 2B6 and 2E1) were studied in both neuronal and glial cell lines exposed to various concentrations of CYP inducers and pesticide-monocrotophos as described in experimental design. The western blot analysis was done following the protocol described earlier by us [49]. In brief,cells were pelleted and lysed using CelLytic™ M Cell Lysis Reagent (Cat No# C2978, Sigma, USA) in the presence of protease inhibitor cocktail (Cat No# P8340, Sigma, USA). Protein estimation was done using the BCA Protein Assay Kit (Cat No# G1002, Lamda Biotech, Inc., St. Louise, MO, USA). Then denatured proteins (100 µg/well) were loaded and electrophorsed using 10% Tricine-SDS gel [51]. Proteins were transferred on polyvinylidene fluoride (PVDF) membrane (Millipore Cat No# IPVH00010, USA) by the wet transfer method at 180 mA current for 3 h. Nonspecific binding was blocked with 5% nonfat dry milk powder in TBST [20 mM Tris-HCl (pH 7.4), 137 mM NaCl, and 0.1% Tween-20] for 2 h at 37°C. After blocking, the membranes were incubated overnight at 4°C with anti-protein primary antibodies specific for CYP1A1, CYP2B6 and CYP2E1 (1∶1000, Chemicon International, USA), in blocking buffer (pH 7.5). The membranes were then incubated for 2 h at room temperature with secondary anti-primary antibody conjugated with horseradish peroxidase (Chemicon International, USA). Then the blots were developed using Super Signal West Fempto Chemiluminescent Substrate™ (Thermo Fisher Scientific, USA) and Bio-Rad Versa Doc™ Imaging System 4000 (Bio-Rad, PA, USA). The densitometry for protein specific bands was done on Gel Documentation System (Alpha Innotech, USA) with the help of Alpha Ease™ FC Stand Alone V.4.0 software. Actin-β was used as an internal control to normalize the data. Xenobiotics induced alterations are expressed in relative term fold change in expression by comparing the data with respective unexposed controls.

### Translational changes (Immunocytochemical localization)

Immunocytochemical localization of CYPs specific proteins was carried out by using anti-primary antibodies following the protocol of Kapoor et al. [14]. Briefly, cells (1×10^4^ cells/well) were allowed to adhere to the surface of eight well chamber slides (Lab Tek, Campbell). Cells were exposed to xenobiotics as described in experimental design. Following exposure, cells were fixed by using 4% paraformaldehyde for 20 minutes and blocked with PBS containing 0.02% Triton-×100 and 0.1% BSA for 2 h to block the non-specific binding sites. Cells were then washed with PBS and incubated with primary antibodies against specific gene proteins, i.e. rabbit anti human CYP1A1, CYP2B6 and CYP2E1 (dilution-1∶500) (Chemicon International, USA) for 2 h at room temperature followed by washing with PBS. Finally, cells were washed with PBS to remove unbound antibody and incubated with TRITC or FITC label secondary antibody for 15–30 min. Cells were visualized under a fluorescent microscope (Nikon Eclipse 80i equipped with Nikon DS-Ri1 12.7 megapixel camera, Japan) and quantification was done by measuring the change in percent area of protein expression with the help of Leica Qwin 500 Image Analysis Software (Leica, Germany).

### Enzyme activity

Following the respective exposures cells were harvested and processed for microsome preparation following the protocol described earlier by us [13]. In brief, cells were scrapped in PBS at 4°C and pelleted by centrifuging at 500×g for 10 min. The cell pellet was resuspended in microsomal dilution buffer containing 0.1% (v/v) glycerol, 0.25 mM protease inhibitors cocktail, 0.01M EDTA and 0.1 mM dithiothreitol. The cells were then sonicated thrice at 15 Hz for 10 seconds each. Following sonication, the cells were again centrifuged at 9000×g for 20 min. The supernatant was then further centrifuged at 105,000×g for 60 min, to isolate the microsomal fraction. The microsomal pellet, thus obtained was then resuspended in microsomal dilution buffer and protein estimation was done by Bradford's Reagent (Fermentas Inc., Maryland, USA). The activity of 7-ethoxyresorufin-O-deethylase (EROD) for CYP1A1, 7-pentoxyresourfin-O-dealkylase (PROD) for CYP2B6, and N-nitrosodimethylamine demethylase (NDMA-d) for CYP2E1 were determined by following the methods described earlier by us [12], [13], [14], [52] using a Perkin Elmer LS 55 Luminescence spectrophotometer.

#### Statistical analysis

The results are expressed as mean and standard error of means (Mean±SE) for at least three experiments. One way ANOVA followed by post hoc Dunnett's test was employed to detect differences between the groups of treated and control. P<0.05 was taken to indicate significant differences.

## *In Silico* studies

### Homology modeling of Aryl Hydrocarbon Receptor (AHR)

The aryl hydrocarbon receptor (AHR) is a ligand-activated transcription factor and has been known as to regulate xenobiotic metabolizing enzymes. Since the crystal structure of the AHR has not been experimentally determined, hereby we created a homology model. The homology modelling of AHR was performed through SWISS-MODEL Workspace web server [53]. The amino acid sequence of AHR protein with a length of 318 amino acids was retrieved from UniprotKb database (Accession No.: P35869). The PDB database by BLAST was searched to identify suitable template protein 3D structure for modelling of AHR. The model was built based on the template protein (PDB: 4F3LA). The homology 3D protein structure model (model_4) of AHR has been developed for this study.

### Molecular docking

The molecular docking and visualization studies were performed using Discovery Studio v3. 5 (Accelrys Inc., USA, 2013) molecular modeling software. For target protein preparation, structure of the AHR homology model (model_4) was developed, while 3D crystal structures of constitutive androstane receptor (CAR) (PDB: 1XVP) and pregnane x receptor (PXR) (PDB: 1ILH) were retrieved from a repository of experimental explicated crystal structure of biological macromolecules available in the PDB database (Brookhaven Protein DataBank, USA) (http://www.rcsb.org/pdb). Initially the protein preparation protocol was used to perform tasks such as inserting missing atoms in incomplete residues, deleting alternate conformations, removing water, standardizing names of the atoms, modeling missing loop regions. The molecular docking studies were performed to generate the active binding poses of candidate compounds in the active site of the receptor by using a LibDock program of Discovery Studio (Accelrys, USA). LibDock uses protein site features referred to as hot spots, consisting of two types (polar and apolar). Then the ligand positions were placed into the polar and the apolar receptor interactions site. Under parameterization step, the MMFF force field was used to minimize the energy of the ligands. The CAESAR (Conformer Algorithm based on Energy Screening and Recursive build-up) method was used to generate the conformations. The Smart Minimiser was used for *in-situ* ligand minimization. All other docking and scoring parameters used were kept at their default settings. The docking program produced several poses with diverse orientations within the defined active site. All the poses have produced different LibDock scores. The best score was taken into account for further study.

## Results

### Cytotoxicity assessment

Both neuronal and glial cells have shown significant alterations in the percent cell viability against all the tested chemicals in a dose dependent manner, when compared with the unexposed control group. However, the variation in response between cell types was not statistically significant, i.e., <10% (Figure 2 A–H). Cells exposed to 3-MC (1–4 µM) have shown no significant reduction in percent cell till 96 h. Whereas, higher concentrations of 3-MC used, i.e., 8 and 10 µM were found to cause a gradual reduction in percent cell viability (25, 51% of control) in neuronal cells at 24 h, which reaches to significant levels at and above 48 h exposure (Figure 2 A & B). CPA concentrations (0.5–2 mM) were found safe in all the exposure periods i.e., 24–96 h. Whereas, higher concentrations of CPA i.e., 4 and 8 mM were found to cause a gradual reduction in percent cell viability, which reaches to significant levels in the exposure period 48 and 96 h (Figure 2 C & D). In general, ethanol exposure was found to be non-cytotoxic for all the exposure periods, except the highest concentration used, i.e., 400 mM for 48, 72 and 96 h in both the cell types (Figure 2 E & F). Though, there was a gradual decrease in the percent cell viability in cells exposed to MCP (10^−7^–10^−5^M) for the period 24–96 h, but it was statistically insignificant. MCP exposure at 10^−4^ and 10^−3^ M was significantly cytotoxic even at 24 h and the magnitude was increased by the extended exposure period, i.e., 48, 72 and 96 h (Figure 2 G & H).

**Figure 2:** Identification of noncytotoxic doses of 3-methylecholentrin (3-MC), cyclophosphamide (CPA), ethanol and known neurotoxicant- monocrotophos (MCP) in neuronal (SH-SY5Y) and glial (U373-MG) cell lines. Cells were exposed to 3-MC (1–10 µM) for 24–96 h in SH-SY5Y (**A**) and U373-MG cells (**B**), CPA (0.5–8 mM) for 24–96 h in SH-SY5Y (**C**) and U373-MG cells (**D**), ethanol (25–400 mM) for 24–96 h in SH-SY5Y (**E**) and U373-MG cells (**F**), and MCP (10^−7^–10^−3^M) for 24–96 h in SH-SY5Y (**G**) and U373-MG cells (**H**). The percent cell viability was assessed using MTT assay. Values are given as mean ± SE of the data obtained from three independent experiments. * = p<0.05, ** = p<0.01.

### Xenobiotics induced transcriptional changes in CYPs

Neuronal cells show a significant gradual increase in the expression of CYP1A1 following the exposure to 3-MC (4 µM) for 1, 3, 6 and 12 h i.e., 2.91±0.35, 4.10±0.17, 7.39±0.78 and 11.96±0.58 fold of control respectively. Cells were also showing significant induction in the expression of CYP1A1 when exposed to MCP for 6 and 12 h; however the magnitude of induction was comparatively lower to that of 3-MC exposed cells. A pre-exposure of 3-MC for 12 h shows the significant additive effect on the up-regulation in the expression of mRNA of CYP1A1 in cells exposed to MCP for 1, 3, 6 and 12 h i.e., 13.29±0.65, 16.19±0.69, 18.89±0.64 and 21.69±0.68 fold of control respectively. The trend of up regulation in the expression of mRNA of CYP1A1 in glial cells was similar to that of neuronal cells; however, the magnitude of expression was a little bit higher than neuronal cells (Figure 3 A & B). Neuronal cells responded significantly against cyclophosphamide (CPA; 2 mM) exposure for 3, 6 and 12 h by inducing the expression levels of mRNA of CYP2B6 (2.67±0.13, 4.38±0.19 and 7.49±0.40 fold of control respectively). Pre-exposure of CPA (12 h) provided an additive response to MCP induced expressions of mRNA of CYP2B6 in neuronal cells. The similar trend and magnitude of induction in the expression levels of mRNA of CYP2B6 was also recorded in glial cells (Figure 3 C & D). Both neuronal and glial cells were also found to induce expression levels of mRNA of CYP2E1 against the exposure of known inducer i.e., ethanol. The pre-exposure of ethanol also found to impose significant additive effect to the response of MCP exposure for 6 and 12 h in both neuronal and glial cells (Figure 3 E & F).

**Figure 3:** Real Time PCR analysis for xenobiotics induced transcriptional changes in CYP genes in SH-SY5Y and U373-MG cells. Fold changes in altered mRNA expression of CYP1A1 in SH-SY5Y cells (**A**) and U373-MG cells (**B**) following the exposure of 3-MC (1–12 h), MCP (1–12 h) and 3-MC (12 h) then MCP (1–12 h) groups. Fold changes in altered mRNA expression of CYP2B6 in SH-SY5Y cells (**C**) and U373-MG (**D**) cells following the exposure of CPA (1–12 h), MCP (1–12 h) and CPA (12 h) then MCP (1–12 h) groups. Fold changes in altered mRNA expression of CYP2E1 in SH-SY5Y cells (**E**) and U373-MG (**F**) cells following the exposure of ethanol (1–12 h), MCP (1–12 h) and ethanol (12 h) then MCP (1–12 h) groups. β-actin was used as endogenous control to normalize the data and xenobiotic exposure induced alterations in transcripts are expressed in fold changes (mean ± SE) compared with unexposed controls. * = p<0.05 and ** = p<0.01 in comparison to respective unexposed controls; while, # = p<0.05 and ## = p<0.01 in comparison to 3-MC, CPA and ethanol (12) exposure respectively.

### Xenobiotics induced translational changes in CYPs

The translational studies carried out using western blot analysis and immunocytochemical localizations have shown the similar trends of induction of CYP 1A1, 2B6 and 2E1 as to that of transcription levels (Figures 4 A–D). In western blot analysis, a gradual induction in the protein expression of CYP1A1 was observed in both neuronal and glial cells exposed to known inducer 3-MC (4 µM) for 24–96 h. MCP exposure could not cause significant induction in level of CYP1A1 at any time point. Whereas, a pre-exposure of 3-MC (12 h) added significantly to the induced levels of CYP1A1 protein in both neuronal and glial cells (Figure 4 A & B). The highest induction of CYP1A1 (3.71 and 4.93 fold of control) was found in neuronal and glial cells, respectively, while receiving pre-exposure of 3-MC followed by the MCP (Figure 4 A & B).

**Figure 4:** Western blot analysis for xenobiotic induced translational changes in CYP proteins in SH-SY5Y and U373-MG cells. (**A**) Western blot analysis of expression of CYP1A1 protein in SH-SY5Y cells following the exposure of 3-MC (24–96 h), MCP (24–96 h) and 3-MC (12 h) followed by post-exposure of MCP (24–96 h). (**B**) Western blot analysis of expression of CYP1A1 protein in U373-MG cells following the exposure of 3-MC (24–96 h), MCP (24–96 h) and 3-MC (12 h) followed by post-exposure of MCP (24–96 h). (**C**) Western blot analysis of expression of CYP2B6 protein in SH-SY5Y cells following the exposure of CPA (24–96 h), MCP (24–96 h) and CPA (12 h) followed by post-exposure of MCP (24–96 h). (**D**) Western blot analysis of expression of CYP2B6 protein in U373-MG cells following the exposure of CPA (24–96 h), MCP (24–96 h) and CPA (12 h) followed by post-exposure of MCP (24–96 h). The values obtained in unexposed cells were considered basal, i.e., relative quantification in expression at different point of various exposures was done comparing the values of unexposed controls. β-actin was used as endogenous control to normalize the data.

CPA exposure induced responses for the CYP2B6 could be observed in both neuronal and glial cells in a time dependent manner with picking values of 1.64 and 2.0 fold of control respectively at 96 h (Figure 4 C & D). Similar to transcriptional changes, there were no significant alterations in the expression of CYP2B6 protein in cells exposed to MCP. Data showed that MCP in presence classical inducers CPA was capable of inducing CYP2B6 in a synergistic way with picking values of 2.96 and 3.70 fold of control in neuronal and glial cells respectively at 96 h (Figure 4 C & D). Data of immunocytochemical localization for CYP1A1 and 2B6 show the linearity with western blot analysis for both neuronal and glial cells and maximum percent area of expression was observed at 96 h (Figure 5 A, B and 6 A, B).

**Figure 5:** Immunocytochemical localization for relative quantification of xenobiotics induced alteration in protein expression of CYP1A1 in SH-SY5Y and U373-MG cells. Changes in % area of expression of CYP1A1 protein in SH-SY5Y cells (**A**) and U373-MG cells (**B**) following the exposure of 3-MC (12–96 h), MCP (24–96 h) and 3-MC (12 h) then MCP (24–96 h) groups. Data are expressed in mean ± SE of percent area of expression in the snapped microscopic fields. A minimum of 20 microscopic fields were snapped for each group. ** = p<0.01 in comparison to respective unexposed controls; while, ## = p<0.01 in comparison to 3-MC (12 h) exposure respectively. Bar indicated in figures = 50 µm.

**Figure 6:** Immunocytochemical localization for relative quantification of xenobiotics induced alteration in protein expression of CYP2B6 in SH-SY5Y and U373-MG cells. Changes in % area of expression of CYP2B6 protein in SH-SY5Y cells (**A**) and U373-MG (**B**) cells following the exposure of CPA (12–96 h), MCP (24–96 h) and CPA (12 h) then MCP (24–96 h) groups. Data are expressed in mean ± SE of percent area of expression in the snapped microscopic fields. A minimum of 20 microscopic fields were snapped for each group. ** = p<0.01 in comparison to respective unexposed controls; while, ## = p<0.01 in comparison to CPA (12 h) exposure respectively. Bar indicated in figures = 50 µm.

The expression of CYP2E1 could not be detected by western blot analysis in any set of experimental or control group. However, ethanol and MCP induced changes in CYP2E1 could be detected in immunocytochemical localization studies. Ethanol (100 mM) induces the significant (p<0.01) expression of CYP2E1 at each point of exposure with peaked expression at 96 h (88±3.87%) in SH-SY5Y cells and U373-MG cells (77±3.35%). In MCP exposed neuronal and glial cells, we could not see the significant alterations in the expression of CYP2E1. However, in ethanol pre-exposed cells MCP showed a synergistic effect in induction of CYP2E1. In ethanol pre-exposed neuronal cells, MCP induces the expression area of 56±3.06% at 24 h, which increases to 97±4.33% area by 96 h, while the glial cells with similar exposure show the highest area of expression 88±3.81% (Figure 7 A & B).

**Figure 7:** Immunocytochemical localization for relative quantification of xenobiotics induced alteration in protein expression of CYP2E1 in SH-SY5Y and U373-MG cells. Changes in % area of expression of CYP2E1 protein in SH-SY5Y cells (**A**) and U373-MG (**B**) cells following the exposure of ethanol (12–96 h), MCP (24–96 h) and ethanol (12 h) then MCP (24–96 h) groups. Data are expressed in mean ± SE of percent area of expression in the snapped microscopic fields. A minimum of 20 microscopic fields were snapped for each group. ** = p<0.01 in comparison to respective unexposed controls; while, ## = p<0.01 in comparison to ethanol (12 h) exposure respectively. Bar indicated in figures = 50 µm.

### Xenobiotics induced alterations in the catalytic activity of CYPs

In general, the microsomal fractions from both neuronal and glial cells show significant induction in CYP dependent EROD (CYP1A1), PROD (CYP2B6) and NDMA-d (CYP2E1) activity. The trend in the induction of CYPs activity was fairly correlated with the data of western blot analysis and real time analysis (Figure 8 A–F).

**Figure 8:** Xenobiotics induced alteration in CYPs specific enzymatic activity in SH-SY5Y and U373-MG cells. EROD (CYP1A1) activity in SH-SY5Y cells (**A**) and U373-MG cells (**B**). Different experimental groups were exposed to 3-MC (12–96 h), MCP (24–96 h) and pre-exposure of 3-MC (12 h) then MCP (24–96 h) exposure. PROD (CYP2B6) activity in SH-SY5Y cells (**C**) and U373-MG cells (**D**). Different experimental groups were exposed to CPA (12–96 h), MCP (24–96 h) and pre-exposure of CPA (12 h)+then MCP (24–96 h) exposure. NMDA-*d* (CYP2E1) activity in SH-SY5Y cells (**E**) and U373-MG cells (**F**). Different experimental groups were exposed to ethanol (12–96 h), MCP (24–96 h) and pre-exposure of ethanol (12 h)+then MCP (24–96 h) exposure. Data are expressed in mean ± SE of specific activity (in their respective units) of catalytic activity in microsomal fractions. * = p<0.05 and ** = p<0.01 in comparison to respective unexposed controls; while, ## = p<0.01 in comparison to 3-MC, CPA and ethanol (12) exposure respectively.

3-MC, a known inducer of CYP1A1 causes significant (p<0.01) induction in the catalytic activity of CYP1A1 (4.12±0.19, 4.96±0.62, 6.73±0.73, 8.49±1.03 and 11.89±1.18 pmoles of resorufin/min/mg protein at 12 h, 24 h, 48 h, 72 h and 96 h, respectively) in neuronal cells while, (3.1±0.16, 3.69±0.39, 5.83±0.59, 7.97±0.68 and 10.15±1.09 pmoles of resorufin/min/mg protein at 12 h, 24 h, 48 h, 72 h and 96 h respectively) in glial cells. MCP alone again failed to activate the CYP1A1 enzyme to catalyze. 3-MC pre-exposure significantly (p<0.01) induces the EROD induction capacity of MCP in both neuronal (Figure 8 A) and glial cells (Figure 8 B).

In case of PROD, the specific activity of CYP2B6 was increased from (5.63±0.53) at 12 h to (14.92±1.34) at 96 h in neuronal cells and from (4.12±0.39) at 12 h to (12.21±1.24) at 96 h in glial cells following the exposure of CPAs. MCP did not induce the activity of CYP2B6 at any time point. CPA pre-exposed neuronal cells show significant induction in the PROD activity upon the exposure of MCP i.e., 8.76±0.74 pmoles of resorufin/min/mg protein at 24 h to 24.48±1.67 pmoles of resorufin/min/mg protein at 96 h. In glial cells, MCP after the pre-exposure of CPA induces CYP2B6 activity at all points of exposure with peak expression at 96 h (20.82±1.40) (Figure 8 C & D).

Ethanol, known inducer of CYP2E1, induces the NDMA-d activity in neuronal cells at each point of exposure, such as at 12 h (2.12±0.10) to 96 h (7.19±0.88). Likewise, in glial cells, ethanol induced increase in specific activity of CYP2E1 has been recorded, i.e., at 12 h (1.8±0.08) and at 96 h (6.45±0.72). MCP could not induce the specific activity of CYP2E1 significant in any cell type used even at any time point of exposure. However, MCP significantly enhances the specific activity of CYP2E1 (NDMA-d) in both neuronal and glial cells pre-exposed to ethanol. The peak induction was observed at 96 h in both neuronal (22.46±1.26) and glial (18.94±0.96) cells respectively (Figure 8 E & F).

### Protein-ligand docking studies

The results of possible mechanisms of action of MCP in relation to human CYP regulators (CAR, PXR and AHR) revealed through molecular docking studies are summarized in Figure 9 (A–E), 10 (A–D), 11 (A–D) and Table 1. The finding demonstrates a significant modulatory activity of MCP to the respective receptors of CYP. This compound exhibited single hydrogen (-H) bonds with each of the studied receptor, i.e., CAR, PXR and AHR. The amino acid residue interacted with MCP through (-H) bond was histidine (HIS-327) of PXR and arginine (ARG-281) & (Arg-316) of AHR and CAR respectively (Table 1). Similarly, the result shows that 3-MC, a highly carcinogenic polycyclic aromatic hydrocarbon, have positive positive interactions with all the three CYP receptors. 3-MC has shown comparatively better docking (LibDock) score than that of other compounds used in this study, i.e., MCP, CPA and ethanol (Table 1). It's LibDock score with CAR receptor CAR was 112.426 and has shown an exposing (-H) bond interaction with tryptophan (TRP-305). MC represents a score of 114.962 through AHR receptor. These scoring are considered as significantly good interaction between compound and receptors. The compound 3-MC has shown a LibDock score of 87.5779 with PXR and presenting Pi-Pi interaction and Pi-sigma interaction with amino acid residue arginine (ARG-410) and methionine (MET-323). This score is also considered to be a good docking score, implies to more effective binding with the receptors and may be a more toxic than other tested compounds. Correspondingly the result for CPA revealed that it can bind more effectively with AHR receptor. This binding represents a LibDock (docking) score of 90.4056 and a single (-H) bond interaction with residue arginine (ARG-281). On the other hand, this compound illustrates a LibDock score of 85.5133 with CAR and 71.5965 with PXR. The amino acid residues involved in the hydrogen bond interactions were leucine (LEU-309) of CAR and arginine (ARG-410) & serine (SER-208) of PXR. Apart this the molecular docking result of ethanol, known inducer of CYP2E1, specifies that it can partially interact with only one of the receptor i.e., CAR. With this receptor its represent a low docking score (LibDock) of 26.835 (Table 1). The amino acid residue involved in these interactions was arginine (ARG-316) and alanine (ALA-327). On the other hand, results indicate that there is no interaction between ethanol and receptors PXR & AHR.

**Figure 9:** Crystal structure of receptors with docked Ligands. (**A**) Crystal structure of CAR (PDB ID: 1XVP) (**B**) Co-crystallized structure of CAR and docked compound monocrotophos (**C**) Co-crystallized structure of CAR and docked compound 3-methylcholanthrene (**D**) Co-crystallized structure of CAR and docked compound Cyclophosphamide (**E**) Co-crystallized structure of CAR and docked compound Ethanol.

**Figure 10:** Crystal structure of receptors with docked Ligands. (**A**) Crystal structure of PXR (PDB ID: 1ILH) (**B**) Co-crystallized structure of PXR and docked compound Monocrotophos (**C**) Co-crystallized structure of PXR and docked compound 3-methylcholanthrene (**D**) Co-crystallized structure of PXR and docked compound Cyclophosphamide.

**Figure 11:** Crystal structure of receptors with docked Ligands. (**A**) Structure of Homology Modeling of Aryl Hydrocarbon Receptor (AHR) Model_4 (**B**) Co-crystallized structure of AHR and docked compound Monocrotophos (**C**) Co-crystallized structure of AHR and docked compound 3-methylcholanthrene (**D**) Co-crystallized structure of AHR and docked compound Cyclophosphamide.

**Table 1:** LibDock scoring, H-Bonding analysis, Pi-sigma interaction and Pi-Pi stacking analysis between candidate compounds and receptors.

S.No.	Compound	Protein Target receptor	LibDock score	H-Bonding analysis	Pi-sigma interaction analysis	Pi-Pi interaction analysis
1 (a)	Monocrotophos	CAR	75.2769	Arg-316	-	-
(b)	Monocrotophos	PXR	64.4324	HIS-327	-	-
(c)	Monocrotophos	AHR	78.1077	ARG-281	-	-
2 (a)	3-methylcholanthrene	CAR	112.426	No-H bonding	-	TRP-305
(b)	3-methylcholanthrene	PXR	87.5779	No-H bonding	MET323	ARG410
(c)	3-methylcholanthrene	AHR	114.962	No-H bonding	-	-
3 (a)	Cyclophosphamide	CAR	85.5133	Leu-309	-	-
(b)	Cyclophosphamide	PXR	71.5965	ARG-410, SER-208	-	-
(c)	Cyclophosphamide	AHR	90.4056	ARG-281	-	-
4 (a)	Ethanol	CAR	26.835	ARG-316, ALA-327	-	-
(b)	Ethanol	PXR	Not docked	-	-	-
(c)	Ethanol	AHR	Not docked	-	-	-

## Discussion

The data of alterations in the expression (mRNA and protein) and marker CYPs enzyme activity in cultured human brain neuronal and glial cells have demonstrated that even at lower doses (non-cytotoxic dose), monocrotophos (MCP) is an inducer of these CYPs. These MCP induced alterations in the expression and activity of different CYP isoforms could be indicative of their metabolism in these cells. Though, the magnitude of induction was not as high as observed in PC12 cells, rat pheochromocytoma cells [49], but reached to the significant levels, when exposed for longer duration. Though, there is no *in vitro* study available dealing with MCP and any other organophosphate pesticide for the expression and activity of CYPs in cultured brain cells, but the trends of time-dependent increase in the expression of CYPs and CYP-dependent enzymatic activity (NDMA-*d*, PROD and EROD) were quite parallel as reported earlier in rat brain exposed to deltamethrin and pyrethroid pesticides [54], [55] and in primary cultures of rat brain neuronal and glial cells [12], [13], [14]. The higher concentrations of MCP (10^−4^M) show the relatively lesser degree of induction of CYPs and CYP associated catalytic activity in both neuronal and glial cells could be attributed due to metabolic accumulation of MCP or its metabolites/enzyme saturation or may be associated with cell mortality [56].

In the present investigations, the MCP induced increase in expression levels and activity of CYPs was not as high as that in the levels induced by classical inducers of CYPs viz., 3-MC (CYP1A1), CPA (CYP2B6), ethanol (CYP2E1). But, MCP is documented as potent developmental neurotoxicant, which inhibits acetylcholine-mediated neurotransmission in the brain [57]. Such inhibitions of neurotransmitter might be associated with MCP induced alterations in the CYPs expression, and thus to the associated neurotoxic effects [49], [57]. Earlier, the association of induced levels of selected xenobiotic metabolizing CYPs has been shown with reactive oxygen species generation and mitochondrial caspase cascade mediated apoptosis in PC12 cells following the exposure of MCP [49], [58]. The activation of CYPs and their interaction with mitochondrial chain complexes in organophosphates-induced apoptosis in neuronal cells have also been reported [59], [60].

Both neuronal (SH-SY5Y) and glial (U373-MG) cells have shown specific and significant response to classical inducers of CYPs viz., 3-MC, CPA and Ethanol by inducing the expression and activity of CYP1A1, 2B6 and 2E1 respectively. The response was quite anticipated and follow the trend as observe earlier in primary cultures of rat brain neuronal and glial cells [12], [13], [14] and in PC12 cells [49]. In the interesting finding, MCP induces alteration in the expression and catalytic activity of CYPs either showing additive responses in both neuronal and glial cells receiving a pre-exposure (12 h) of known inducer i.e., 3-MC/CPA/Ethanol. Such additive effect of MCP to the expression and activity of all the three CYPs studied in pre-sensitized cells indicate the involvement of all these CYPs in the metabolism of MCP. The findings also indicate that non-sensitized cells were not having enough triggering signals to induce the expression and activity like primary cultures of rat brain neuronal and glial cells [14] and in PC12 cells [49]. Thus, the findings suggest the xenobiotic metabolizing capabilities of these cells against MCP or may be to any other organophosphate pesticide, provided they received a pre-sensitization stimulus to trigger the xenobiotic metabolizing machinery in them. It is widely documented that the specific chemicals contributes significantly to induce the expression of specific xenobiotic metabolizing enzymes by inducing the increased expression of the master regulators of CYPs genes viz., aryl hydrocarbon receptor (AHR), constitutive androstane receptor (CAR) and pregnane-X-receptor (PXR) [61]. In the present investigation, it seems that MCP profoundly adds/synergizes classical CYP-inducers viz., 3-MC, CPA and ethanol (ligands of AHR, CAR and PXR) in inducing the expression of CYP1A1, 2B6 and 2E1 respectively. Thus, MCP might be trans-activating these master regulators of CYPs (AHR, CAR and PXR).

The linearity in the expression and inducibility between mRNA and protein level (Western blot analysis) for CYP2E1 could not be established. While, the trends were similar for mRNA and immunocytochemical localization and catalytic activity in case of CYP2E1. Such inconsistency might be due to the post-translational regulation of CYP2E1, which involves various cellular factors viz., insulin, growth hormones, epidermal growth factor, etc. [35]. Besides that, the mechanism of CYP2E1 induction is complex, depends on the substrate, species, tissue, or cell type [35], [36], [37]. Several levels of gene regulation like transcription, translation, and post-translational modification, play an important role in maintaining the proper function of CYPs. Post-translational modifications (like phosphorylation, glycosylation, nitration), ubiquitination for proteasome mediated protein degradation, targeting to specific cellular compartments are well reported for non-consistency between the expression of mRNA and the protein of CYPs [62]. Recently, CYPs and their nuclear receptor regulators have been found to be post-transcriptionally regulated by miRNAs. Mohri et al., [63] reported that the molecular mechanism of CYP2E1 regulation by miR-378 to clarify the non-consistency between mRNA and protein expression of CYP2E1.

The ability of MCP to induce the expression of neuronal CYPs is of significance as studies have indicated a role of CYPs in neurotransmission [64]. Studies have also shown that modulation in the activity of brain CYPs affects neurotransmission altering either synthesis or transport of neurotransmitters [65]. Possible endogenous substrates for CYP1A1, 2B6 and 2E1 have also been identified in the brain [66]. CYP2E1 has been associated with dopaminergic neurotransmission; the enhanced expression of neuronal CYP2E1, in particular could be attributed to the dopaminergic effect of MCP. Kirby et. al., [67] have earlier reported that pesticide treated in combination with MPTP, a parkinsonian neurotoxin, caused a significant increase in dopamine uptake, consistent with the increased dopamine outflow *in vivo* and suggested an up-regulation in the dopamine transporter expression. Though, the exact mechanism of pesticides, including organophosphates, in the etiology of Parkinson's disease (PD) remains to be established. Franco et al., [68] have reported that low level exposure to organophosphates may contribute to PD through up-regulation of dopamine transporter and increased uptake of endogenous and exogenous neurotoxicants while increased levels result in apoptotic cell death. Thus, considering that CYP2E1 has a role in dopamine metabolism [65], and the fact that CYP2E1 has been found to be co-localized with tyrosine hydroxylase [69], one could speculate that the MCP induced alterations in neuronal CYP2E1 could, in turn, be associated with alterations in the levels of dopamine induced by the MCP.

The increase in the activity of CYP1A1 and CYP2B6 isoforms, in cultured neurons following MCP exposure could also be of significance, as earlier studies from our laboratory have shown the involvement of these xenobiotic metabolizing CYPs in the neurobehavioral toxicity of pyrethroid pesticide-deltamethrin [70]. The increase in the expression of these CYPs in cultured neurons on exposure to MCP could also be associated with the alterations in the specific brain functions catalyzed by these cells, as well as by these CYP isoforms. The specific increase in the expression of CYP1A1, in MCP exposed cultured neurons could be associated with the alterations in the levels of catecholamines. Organophosphates have been earlier reported to alter the levels of various catecholamines in different brain regions [71]. The concentrations of acetylcholine were found to be altered in the cerebellum and hippocampus and that of dopamine in the striatum [72]. Studies have indicated that catecholamines and adrenoreceptors are involved in the regulation of CYP1A1 expression [73]. A relation between neurological effects of barbiturates mediated via binding with GABA receptor complex, and their capacity to induce CYP2B proteins have been reported [32]. Studies using reporter gene protocol have also shown that ligands of peripheral benzodiazepine receptor (PBR) or GABA_A_ receptor induce CYP2B activity, and it was mediated through the PBRU and the nuclear receptor binding sites NRI/NR2 [32].

The induction of CYPs in the expression and catalytic activity of CYP1A1, 2B6 and 2E1 in glial cells is of toxicological significance, as these cells are the main cellular components of the blood-brain barrier (BBB) and have an important physiological role in integrating neuronal inputs, neurotransmitter release and the protection and repair of nervous tissue. Earlier studies have further suggested that astroglial cells play a protective and decisive role in the biotransformation of xenobiotics that reach the CNS [74], [75]. The role of astrocytes in the defense against reactive oxygen species (ROS) has also been reported [76]. Glutathione-S-transferase, the phase II enzyme has also been reported to be localized exclusively in glial cells, constituting a first line of defense against toxic substances [77]. Meyer et. al., who studied the role of astrocyte CYP in the metabolic degradation of phenytoin, observed that CYPs in astrocytes fulfill a mediatory detoxification function by degrading phenytoin to keep the drug response of the neurons in balance [74]. They reported that at high concentration of phenytoin, cytotoxic effects in both neurons and glia interfere with the intended therapeutic action, indicating that the viability of astrocytes and in direct consequence, neurons is negatively affected. Hagemeyer et. al., [78] have also suggested CYP expression in astrocytic population, smooth muscle cells covering micro vessels, in ependymal cells in the choroids plexus, may be involved in protecting the brain from a broad spectrum of neurotoxicants. The greater responsiveness of CYP1A1 and CYP2B6 isoenzymes in glial cells to MCP could be attributed to the involvement of these isoforms in toxication-detoxication mechanisms. However, as CYP1A1 and 2B6 enzyme induction has been found to be correlated with the potentiation of the neurobehavioral toxicity of pyrethroid pesticides, increase in the expression of these isoenzymes in both glial and neuronal cells, could also be involved in the metabolic activation of the organophosphate pesticides such as MCP at the target site(s).

In summary, the expression of CYP1A1, CYP2B6 and CYP2E1 in cultured human neuronal (SH-SY5Y) and glial (U373-MG) cells has suggested that the constitutive expression of these CYPs may possibly be associated with the endogenous physiology of the brain. The increase in the CYPs specific activity and associated expression (mRNA and protein) in cultured neuronal cells induced by MCP could help in explaining its effect on neurotransmission, as these CYPs are involved in the synthesis or transport of the neurotransmitters. Likewise, the induction of CYPs in glial cells is also of significance as these cells are thought to be involved in protecting the neurons from environmental insults and safeguard them from toxicity. The responsiveness of both the cells against MCP exposure enhanced/synergized due to a pre-sensitization with classical inducers of CYPs viz., 3-MC, CPA and ethanol. The *in silico* studies have suggested that three major factors such as (-H) bonding interactions, Pi-sigma interactions and Pi stacking are responsible for the activity of the respective receptors and the candidate compounds. 3-MC can modulate the activity of the CAR and AHR receptors with higher frequency than the other compounds tested. The study provides a better understanding of xenobiotic metabolizing capability of the human brain cells, which will be useful in adopting them for routine neurotoxicity research. At the same time, the precise knowledge of the specific regulatory properties of both glial and neuronal cell lines derived from human brain will give us insights in the understanding the role of CYPs in the toxication/detoxification processes for either environmental pollutants and drugs or endogenous toxins involved in the etiology of neurodegenerative diseases and development/management of therapeutic intervention strategies.

## Supporting Information

Table S1 **Statistical analysis of xenobiotics induced changes in CYP1A1 gene in SHSY-5Y and U373-MG cells.** (a): Real Time PCR analysis of transcriptional changes; (b): Western blot analysis of translational changes; (c): Immunocytochemical localization for relative quantification of protein expression; (d): EROD (CYP1A1) activity.
(DOC)

Table S2 **Statistical analysis of xenobiotics induced changes in CYP2B6 gene in SHSY-5Y and U373-MG cells.** (a): Real Time PCR analysis of transcriptional changes; (b): Western blot analysis of translational changes; (c): Immunocytochemical localization for relative quantification of protein expression; (d): PROD (CYP2B6) activity.
(DOC)

Table S3 **Statistical analysis of xenobiotics induced changes in CYP2E1 gene in SHSY-5Y and U373-MG cells.** (a): Real Time PCR analysis of transcriptional changes; (b): Immunocytochemical localization for relative quantification of protein expression; (c): NDMA*-d* (CYP2E1) activity.
(DOC)
